The article "miR-331-3p Inhibits Proliferation and Promotes Apoptosis of Nasopharyngeal Carcinoma Cells by Targeting elf4B-PI3K-AKT Pathway" was retracted in 2022. Reasons: duplicated images; unreliable results or conclusions.

# miR-331-3p Inhibits Proliferation and Promotes Apoptosis of Nasopharyngeal Carcinoma Cells by Targeting elf4B-PI3K-AKT Pathway

**DOI:** 10.1177/1533033819892251

**Published:** 2020-01-26

**Authors:** Zhang Xuefang, Zheng Ruinian, Jiang Liji, Zhang Chun, Zheng Qiaolan, Jia Jun, Chen Yuming, Huang Junrong

**Affiliations:** 1 Department of Radiotherapy, Dongguan People’ Hospital, Dongguan, China; 2 Department of Medical Oncology, Dongguan People’ Hospital, Dongguan, Guangdong, China; 3 Department of Journal Center, Third Affiliated Hospital of SUN YAT-SEN University, Guangzhou, China

**Keywords:** nasopharyngeal carcinoma, miRNA-331-3p, elF4B, PI3K–AKT signaling pathway

## Abstract

**Background:**

The incidence of nasopharyngeal carcinoma is increasing gradually, but the pathogenesis is not completely clear. MicroRNA, a highly conserved endogenous noncoding small molecule RNA, plays an essential role in the regulation of gene expression and is a hotspot in cancer research worldwide.

**Objectives:**

Although previous studies have confirmed that the abnormal expression of microRNAs is closely related to the progression of nasopharyngeal carcinoma, the role of miRNA-331-3p in nasopharyngeal carcinoma has not been studied. The purpose of this study was to explore the role and mechanism of miRNA-331-3p in the progression of nasopharyngeal carcinoma.

**Materials and Methods:**

Real-time quantitative reverse transcription polymerase chain reaction was performed to detect the expression of miRNA-331-3p in nasopharyngeal carcinoma clinical samples and cell lines (CNE-1 and 5-8F cells). After overexpression of miRNA-331-3p in CNE-1 cells, cell proliferation was measured by Cell Counting Kit-8 assay, cell invasion was detected by Transwell assay, and apoptosis was tested by flow cytometry. In addition, the dual-luciferase reporter assay was used to identify the target gene of miRNA-331-3p and Western blotting was performed to measure the relative protein expression.

**Results:**

The expression of miRNA-331-3p in nasopharyngeal carcinoma clinical samples and cells was decreased significantly. Overexpression of miRNA-331-3p markedly inhibited the proliferation and invasion of CNE-1 cells and promoted cell apoptosis. Moreover, overexpression of miRNA-331-3p reduced the expression of target gene elF4B, leading to inhibition of the phosphorylation of Phosphoinositide 3-kinase (PI3K) and Serine/ threonine kinase (AKT).

**Conclusion:**

miRNA-331-3p inhibited cell proliferation and induced cell apoptosis in nasopharyngeal carcinoma by targeting *elF4B* gene and then blocked the PI3K-AKT signaling pathway.

**Significance:**

The role of miRNA-331-3p in the development of NPC and its mechanism provide new ideas for the treatment of nasopharyngeal carcinoma.

The article "miR-331-3p Inhibits Proliferation and Promotes Apoptosis of Nasopharyngeal Carcinoma Cells by Targeting elf4B-PI3K-AKT Pathway" was retracted in 2022. Reasons: duplicated images; unreliable results or conclusions.

## Introduction

Nasopharyngeal carcinoma (NPC) is a common malignant tumor of the head and neck, and its incidence is closely related to regional distribution.^1^ As there is no obvious clinical symptom in the early stage, most patients with NCP were found in the middle and late stages of the disease, leading to a bad quality of life of people.^2,3^ Nasopharyngeal carcinoma has a strong ability of invasion and metastasis.^4^ Distal metastasis is a common feature of NPC. Thus, controlling its metastasis is the key factor in the treatment of NPC.^4,5^ At present, radiotherapy and chemotherapy are mostly used in the treatment of NPC, which has a low 5-year survival rate and unsatisfactory effect.^6^ The etiology of NPC is not yet clear. It is generally believed to be associated with heredity, viral infection, and environmental factors.^7,8^ Therefore, searching for molecular targets related to the pathogenesis and progression and exploring relevant mechanisms are of great significance for the early diagnosis and treatment of NPC.

MicroRNA (miRNA) is a highly conserved endogenous noncoding small molecule RNA with a length of about 18 to 21 nucleotides.^9^ It participates in many biological processes through complex biological regulatory networks in organisms.^9,10^ MicroRNA binds to the noncoding regions of target genes in a way of incomplete complementary pairing and inhibition of the synthesis of target genes and thus regulating cell proliferation, individual metabolism, and development.^9-11^ In recent years, numerous studies have proved that miRNA is closely related to tumorigenesis, including occurrence, invasion, and metastasis.^12,13^ Some miRNAs such as miRNA-135b,^14^ miRNA-182,^14^ and miR-346^15^ have an enhancing effect on cell proliferation and metastasis in NPC, while some miRNAs such as miR-223,^16^ miRNA-29,^13,17^ and miR-200a^18^ induce apoptosis and prohibit the progression of NPC.

miRNA-331-3p, a member of the family of miRNAs, has an essential effect on the occurrence and development of multiple tumors.^19^ It is considered to be a tumor-related factor, which participates in the progression of tumors by targeting genes.^20,21^ Zhao *et al*^22^ have shown that miRNA-331-31p suppresses proliferation and enhances apoptosis in colorectal cancer. De Martino *et al*^19^ reported that miRNA-331-3p exerts influence on the regulation of the development of cancer by modulating High mobility group protein A1 pathway. These studies suggest that miRNA-331-3p may be a new target for cancer therapy, but there are few reports on NPC at present. In the present study, we investigated the expression of miRNA-331-3p in NPC and further explored its target gene and molecular mechanism, which may provide novel targets for the treatment of NPC.

The article "miR-331-3p Inhibits Proliferation and Promotes Apoptosis of Nasopharyngeal Carcinoma Cells by Targeting elf4B-PI3K-AKT Pathway" was retracted in 2022. Reasons: duplicated images; unreliable results or conclusions.

## Materials and Methods

### Human Tissue Samples

Nasopharyngeal carcinoma tissues and normal adjacent tissues (60 cases each) were obtained from the Radiotherapy Department of Dongguan People’s Hospital. The written informed consent of every patient was required. The study was approved by the Medical Ethics Committee of Dongguan People’s Hospital.

### Cell Culture

Nasopharyngeal epithelial cells NP69 were maintained in K-SFM medium (Gibco, Grand Island, New York) without serum growth factor. Nasopharyngeal carcinoma cell lines 5-8F and CNE-1 were cultured in RPMI-1640 medium (Gibco) with 10% fetal bovine serum (Gibco). All 3 cells were grown in the incubator at 37°C with 5% CO_2_. Cells were fused to 70% to 80% and passaged for subsequent experiments.

### Cell Transfection

CNE-1 cells were inoculated into a 6-well plate at a density of 10^5^. Then cells were transfected with microRNA-331-3p mimic with Lipo 3000 (RiboBio, Guangzhou, China). Small interfering RNA duplexes with nonspecific sequences were used as the negative control (NC). After transfection for 48 hours, cells were collected for subsequent experiments.

### Cell Proliferation Assay

CNE-1 cells were plated in a 96-well plate with a density of 10^3^. After 24, 48, and 72 hours of culture, a Cell Counting Kit-8 (CCK-8; Dojindo, Kumamoto, Japan) was used to detect the cell proliferation in the light of manufacturer’s instructions. The absorbance value was measured at 450 nm.

### Cell Invasion Assay

Treated cells were cultured in the Transwell chamber with Matrigel-coated membrane (BD Biosciences, Bedford, Massachusetts). After 24 hours of culture, cells were fixed with 4% paraformaldehyde (Servicebio, Wuhan, China). After that, the cells were stained with crystal violet and washed 3 times with phosphate-buffered saline (PBS). Five visual fields were selected for counting under the microscope.

### Cell Apoptosis Assay

CNE-1 cells were plated in a 6-well plate with a density of 10^5^. After 48 hours of culture, cells were collected and resuspended in 100 μL buffer. Then cells were stained with Annexin V- Fluoresceine isothiocyanate and propidium iodide for 15 minutes on ice. Cells were cleaned twice with precooled PBS and then the apoptotic rate was measured using the CytExpert software (Beckman-Coulter, Miami, Florida).

### Dual-Luciferase Reporter Assay

miR-Base (http://www.mirbase.org/) and TargetScan Human 7.0 (http://www.targetscan.org/) microRNA databases were used to predict the target gene of miRNA-331-3p. Wild-type and mutated elF4B-3′-untranslated region (UTR) sequence (containing mutated binding sites of miRNA-331-3p) was amplified by polymerase chain reaction and cloned into pGL3 Basic Vector (Promega, Madison, Wisconsin), respectively. Then 293 cells were cotransfected with reporter vectors and miR-331-3p mimic. The luciferase activity was measured using the dual-luciferase reporter assay system.

The article "miR-331-3p Inhibits Proliferation and Promotes Apoptosis of Nasopharyngeal Carcinoma Cells by Targeting elf4B-PI3K-AKT Pathway" was retracted in 2022. Reasons: duplicated images; unreliable results or conclusions.

### Real-Time Quantitative Reverse Transcription Polymerase Chain Reaction

Total RNA was extracted from CNE-1 cells using TRIzol reagent (Invitrogen Life Technology, Carlsbad, California). PrimeScript RT reagent kit (Takara, Shiga, Japan) was used to reverse transcribe RNA into complementary DNA, which was used for the following quantitative reverse transcription polymerase chain reaction (RT-qPCR) analyses by the SYBR Premix Ex Taq II (Tli RNaseH Plus) kit (Takara). Vii7 System (Applied Biosystems, Waltham, Massachusetts) was used to quantify and analyze messenger RNA.

### Western Blotting

The protocol used for protein quantification was described in a previous study.^23^ The antibodies used were as follows: rabbit anti-elF4B, anti-p-Serine/ threonine kinase (AKT), anti-AKT (CST), anti-p-Phosphoinositide 3-kinase (PI3K), anti-PI3K, anti-B-cell lymphoma-2 (Bcl-2), anti-Bcl-2-associated X protein (Bax), anti-caspase-3/c-caspase-3, anti-caspase-9/c-caspase-9, anti-glyceraldehyde-3-phosphate dehydrogenase, and anti-rabbit immunoglobulin G. All antibodies were obtained from Cell Signaling Technology (Beverly, Massachusetts) and Santa Cruz Biotechnology (Santa Cruz, California).

### Statistical Analysis

The data are presented as the mean ± standard deviation. Student *t* test was performed for comparison of statistical difference between 2 groups and one-way analysis of variance for more than 2 groups by SPSS 22.0 (IBM Inc, Chicago, Illinois). Statistical significance was established at *P* value <.05.

## Results

### Downregulation of miRNA-331-3p in NPC Tissues and Cells

Quantitative reverse transcription polymerase chain reaction was performed to detect the RNA expression of miRNA-331-3p in 60 NPC tissues and matched normal tissues. The results showed that the expression of miRNA-331-3p in NPC tissue was significantly lower than that in normal tissues (Figure 1A). Then we tested the RNA level of miRNA-331-3p in NPC cells and normal nasopharyngeal epithelial cells *in vitro*. As depicted in Figure 1B, compared with NP69 cells, the RNA expression of miRNA-331-3p in 5-8F and CNE-1 cells was decreased obviously. All the above findings indicated a downregulation of miRNA-331-3p in NPC tissues and cells.

**Figure 1.** Downregulation of miRNA-331-3p in nasopharyngeal carcinoma (NPC) tissues and cells. A, The RNA expression of miRNA-331-3p in NPC tissues and matched normal tissues (n = 60). B, The RNA expression of miRNA-331-3p in 5-8F, CNE-1, and NP69 cells. Data are shown as the means ± standard deviations. *P < .05, **P < .01.

The article "miR-331-3p Inhibits Proliferation and Promotes Apoptosis of Nasopharyngeal Carcinoma Cells by Targeting elf4B-PI3K-AKT Pathway" was retracted in 2022. Reasons: duplicated images; unreliable results or conclusions.

### Inhibition of Proliferation and Invasion of CNE-1 Cells by miRNA-331-3p

To further explore the action of miRNA-331-3p in NPC cells, we detected the proliferation, invasion, and apoptosis of CNE-1 cells following miRNA-331-3p overexpression. As shown in Figure 2A, overexpression of miRNA-331-3p remarkably inhibited the invasion of CNE1 cells. The results of the CCK-8 assay showed that miRNA-331-3p restrained the cell viability (Figure 2B). We also found that after overexpression of miRNA-331-3p in CNE-1 cells, the expression of vimentin decreased and E-cadherin increased (Figure 2C).

**Figure 2.** miRNA-331-3p inhibits the proliferation and invasion of CNE-1 cells. CNE-1 cells were transfected with microRNA-331-3p mimic, and those transfected with small interfering RNA duplexes with nonspecific sequences were used as the negative control (NC). A, Cell invasion was detected using Transwell invasion assay. B, Cell viability was measured using Cell Counting Kit-8 (CCK-8) assay at 0, 24, 48, and 72 hours of culture. C, The protein expression of vimentin and E-cadherin was detected by Western blot. Data are shown as the means ± standard deviations. *P < .05, compared to control or NC.

### Promotion of Apoptosis in CNE-1 Cells by miRNA-331-3p

Next, we investigated the effect of miRNA-331-3p on apoptosis of CNE-1 cells. Firstly, we detected the apoptotic rate by flow cytometry. As shown in Figure 3A, the apoptotic rate of CNE-1 cells in miR-331-3p overexpression group increased by 2.11 folds compared with that in the control group and 2.53 folds compared with that in the NC group. Then we measured the expression of apoptotic protein, such as poly(adenosine diphosphate-ribose) polymerase (PARP), caspase3, caspase9, Bcl-2, and Bax. The findings showed that miRNA-331-3p upregulated the expression of PARP, caspase3, caspase9, and Bax and downregulated the expression of Bcl-2. These results demonstrated the enhancing effect of miRNA-331-3p on apoptosis of CNE-1 cells (Figure 3B).

**Figure 3.** miRNA-331-3p promotes the apoptosis of CNE-1 cells. CNE-1 cells were transfected with miRNA-331-31p and those transfected with small interfering RNA duplexes with nonspecific sequences were used as the negative control (NC). A, Cell apoptotic rate was measured using flow cytometry. B, The protein expression of poly(adenosine diphosphate-ribose) polymerase (PARP), caspase3, caspase9, B-cell lymphoma-2 (Bcl-2), and Bcl-2 associated X protein (Bax) was detected by Western blot. Data are shown as the means ± standard deviations. *P < .05, **P < .01, compared to control or NC.

The article "miR-331-3p Inhibits Proliferation and Promotes Apoptosis of Nasopharyngeal Carcinoma Cells by Targeting elf4B-PI3K-AKT Pathway" was retracted in 2022. Reasons: duplicated images; unreliable results or conclusions.

### Identification of Target Gene *elF4B* of miR-331-3p

Using TargetScan and miR-Base databases, we predicted that *elF4B* is the downstream regulatory target gene of miR-331-3p, which was verified by the dual-luciferase reporter assay. As shown in Figure 4A, miR-331-3p reduced the luciferase activity of wild-type elF4B-3′-UTR but had no significant effect on the mutant elF4B-3′-UTR. Also, the results of RT-qPCR and Western blotting depicted that miR-331-3p significantly decreased the RNA and protein expression of elF4B (Figure 4B).

**Figure 4.** *elF4B* is a target gene of miR-331-3p. CNE-1 cells were transfected with miRNA-331-31p and those transfected with small interfering RNA (siRNA) duplexes with nonspecific sequences were used as the negative control (NC). A, Sequence of potential binding site of miR-331-3p in the 3′-untranslated region (UTR) of elF4B messenger RNA (mRNA). B, miRNA-331-31p suppressed the luciferase activity of elF4B 3′-UTR but had no significant effect on the luciferase activity of the mutant. C, The mRNA expression of elF4B. D, The protein expression of *elF4B*. Data are shown as the means ± standard deviations. *P < .05, compared to control or NC.

### Regulation of Physiological Function by miR-331-3p via the elF4B-PI3K-Akt Pathway

Next, we explored the possible molecular mechanisms underlying the regulation of physiological functions of miRNA-331-3p. PI3K-AKT pathway has been reported to involve in the regulation of the progression of cancers.^24^ Thus, we investigated whether miRNA-331-3p affects the activation of the PI3K-AKT pathway. We found that miRNA-331-3p markedly suppressed the phosphorylation of PI3K and AKT (Figure 5). Consistently, we observed downregulation of miRNA-331-3p and upregulation of elF4B, phospho-PI3K, and phospho-AKT in NPC tissues (Supplementary Figure 1). These results suggested that miRNA-331-3p may act through the elF4B-PI3K-AKT pathway.

**Figure 5.** miR-331-3p suppresses PI3K-AKT pathway. CNE-1 cells were transfected with the miRNA-331-31p and those transfected with siRNA duplexes with nonspecific sequences were used as the negative control (NC). A, The phosphorylation of AKT was detected by Western blot. B, The phosphorylation of PI3K was detected by Western blot. Data are shown as the means ± standard deviations. **P < .01, compared to control or NC.

## Discussion

In this study, we found that the expression of miRNA-331-3p in NPC tissues and CNE-1 cells was decreased significantly compared with the control group. Overexpression of miRNA-331-3p in CNE-1 cells inhibited the expression of elF4B, thus inactivating the PI3K-AKT pathway, which led to the inhibition of proliferation and invasion of CNE-1 cells. Our results demonstrated that miRNA-331-3p had a vital role in the development of NPC.

The article "miR-331-3p Inhibits Proliferation and Promotes Apoptosis of Nasopharyngeal Carcinoma Cells by Targeting elf4B-PI3K-AKT Pathway" was retracted in 2022. Reasons: duplicated images; unreliable results or conclusions.

Recently, many studies pay attention to NPC because of its increasing incidence, but the pathogenesis of NPC is still unclear.^1^ At the same time, there are more and more studies on the effect of miRNA on the progression of NPC.^25,26^ Overexpression of microRNA-135b enhances the invasion and metastasis ability of CNE1 cells, while downregulation of microRNA-135b expression effectively inhibits the proliferation and promoted the apoptosis of CNE-1 cells, which may be related to the effects on LATS2 activity.^26^ Qi *et al*^27^ indicate that miRNA-142-3p significantly advances the cell proliferation in NPC by inhibiting the expression of target protein SOCS6. miR-29a/b enhances cell migration and invasion via regulation of SPARC and COL3A gene level, which lead to the promotion of the development of NPC.^28^

miRNA-331-3p participates in tumorigenesis and development by regulating downstream target genes, which has attracted increasing attention.^21,29^ miRNA-331-3p is considered as a tumor suppressor gene, which is downregulated in gastric cancer cells,^29^ prostate cancer cells,^30^ pancreatic cancer cells,^20^ cervical cancer cells,^31^ and glioblastoma cells.^32^ However, Chang *et al*^33^ have reported that hepatitis B virus promotes the expression of miRNA-331-3p in hepatocellular carcinoma cells by enhancing promoter activity. miRNA-331-3p may be used as a potential prognostic marker and a novel therapeutic target, but there are few studies on the role of miRNA-331-3p in NPC. In our study, we found that the expression of miRNA-331-3p was significantly downregulated in clinical tissue samples of patients with NPC and NPC cells, which was consistent with the expression of miRNA-331-3p in most cancer cells. Overexpression of miRNA-331-3p inhibited the proliferation and invasion of CNE-1 cells and promoted apoptosis of CNE-1 cells, which were consistent with the results reported in colorectal cancer cells.^22^ Our results suggested that miRNA-331-3p plays an antineoplastic role in the progression of NPC.

miRNA performs biological functions via the regulation of downstream target genes. Presently, we confirmed elF4B as a target gene of miRNA-331-3p by dual-luciferase reporter assay. Gene elF4B interacts with elF4A to enhance the activity of their unwinding RNA and protein elF4B promotes cell proliferation and regulates cell survival through PI3K-AKT pathway. Phosphorylation levels of PI3K and AKT affect the proliferation, invasion, and apoptosis of cancer cells remarkably.^14,22,24^ Yang *et al*^24^ found that miRNA-122 suppresses the expression of TRIM29 and then blocks the activation of PI3K-AKT pathway, which results in the inhibition of the development of NPC. miRNA-148a restrains cell growth of papillary thyroid cancer by relating PI3K-AKT pathway.^34^ In the present study, the protein expression of elF4B and phosphorylation of PI3K and AKT were decreased significantly after overexpression of miRNA-331-3p, indicating that miRNA-331-3p may regulate downstream biological actions via elF48-PI3K-AKT signaling pathway.

The article "miR-331-3p Inhibits Proliferation and Promotes Apoptosis of Nasopharyngeal Carcinoma Cells by Targeting elf4B-PI3K-AKT Pathway" was retracted in 2022. Reasons: duplicated images; unreliable results or conclusions.

In summary, our study showed that the expression of miRNA-331-3p was downregulated in NPC tissues and cells, indicating its significant role in the progression of NPC. Moreover, we found that miRNA-331-3p inhibits the proliferation and invasion and induces apoptosis of CNE-1 cells by blocking elF4B-PI3K-AKT signaling pathway. The molecular mechanism explored in this study may provide a theoretical basis for the pathogenesis of NPC and new molecular targets for the treatment of NPC.

## Supplemental Material

Supplemental Material, Ethical_review - miR-331-3p Inhibits Proliferation and Promotes Apoptosis of Nasopharyngeal Carcinoma Cells by Targeting elf4B-PI3K-AKT Pathway Click here for additional data file. Supplemental Material, Ethical_review for miR-331-3p Inhibits Proliferation and Promotes Apoptosis of Nasopharyngeal Carcinoma Cells by Targeting elf4B-PI3K-AKT Pathway by Zhang Xuefang, Zheng Ruinian, Jiang Liji, Zhang Chun, Zheng Qiaolan, Jia Jun, Chen Yuming and Huang Junrong in Technology in Cancer Research & Treatment

Supplement - miR-331-3p Inhibits Proliferation and Promotes Apoptosis of Nasopharyngeal Carcinoma Cells by Targeting elf4B-PI3K-AKT Pathway Click here for additional data file. Supplement for miR-331-3p Inhibits Proliferation and Promotes Apoptosis of Nasopharyngeal Carcinoma Cells by Targeting elf4B-PI3K-AKT Pathway by Zhang Xuefang, Zheng Ruinian, Jiang Liji, Zhang Chun, Zheng Qiaolan, Jia Jun, Chen Yuming and Huang Junrong in Technology in Cancer Research & Treatment

## Abbreviations

Bcl-2: B-cell lymphoma-2
Bax: Bcl-2-associated X protein
CCK-8: Cell Counting Kit-8
miRNA: microRNA
NC: negative control
NPC: nasopharyngeal carcinoma
PARP: poly(adenosine diphosphate-ribose) polymerase
PBS: phosphate-buffered saline
RT-qPCR: quantitative reverse transcription polymerase chain reaction
UTR: untranslated region
